The article "Effects of Tea Treatments against High-Fat Diet-Induced Disorder by Regulating Lipid Metabolism and the Gut Microbiota" was retracted in 2023. Reasons: unreliable results or conclusions; concerns about the data; concerns about the peer review; concerns about the citations.

# Effects of Tea Treatments against High-Fat Diet-Induced Disorder by Regulating Lipid Metabolism and the Gut Microbiota

**DOI:** 10.1155/2022/9336080

**Published:** 2022-05-29

**Authors:** Chen Wang, Jiaxing Liu, Siyao Sang, Xue Ao, Mingjie Su, Binwei Hu, Hui Li

**Affiliations:** ^1^MOE Key Laboratory of Contemporary Anthropology, Human Phenome Institute, Fudan University, Shanghai 200438, China; ^2^State Key Laboratory of Genetic Engineering, School of Life Sciences, Fudan University, Shanghai 200438, China; ^3^Shanxi Academy of Advanced Research and Innovation, Fudan-Datong Institute of Chinese Origin, Datong 037006, China

## Abstract

High-fat diet (HFD) may induce changes of metabolism and gut microbiota changes, and these changes are susceptible to diet adjustments such as tea treatment. However, the treatment effects may vary among different types of tea. In this study, we evaluated the effects of six types of tea on glucose and lipid metabolism and gut microbiota in HFD mice. We established HFD mouse model by 12 weeks feed with 60% fat diet, then treated with teas for six weeks. Here, we showed that treatment with different types of tea can inhibit weight gain and insulin resistance though different ways. Green tea regulated lipid metabolism by regulating the expression of adenosine 5′-monophosphate-activated protein kinase (AMPK) and carnitine palmitoyltransferase-I (CPT-1). The effect of dark tea and white tea in reducing liver weight seemed to be related to activities of acetyl-CoA carboxylase (ACC). Yellow tea exhibited the best anti-inflammatory and antioxidant effects and effects of recovering the disorder of model mouse microbiota. The decrease in blood sugar and the upregulation of gluconeogenesis-related enzymes seemed to be related to the decrement of unclassified Lachnospiraceae. These different effects may result from the unique chemical compositions contained by different types of tea, which can regulate different lipid and glucose metabolism-related proteins. Despite variations in its compositions and metabolic reactions, tea is a potent antiobesity and hypoglycemic agent.

## 1. Introduction

Excessive dietary fats can result in disorders of glycose and lipid metabolism and gut microbiota and further give rise to negative health impacts including obesity, insulin resistance, diabetes, and nonalcohol fatty liver disease (NAFLD) [1, 2]. Generally, the majority of the excessive energy from diet is stored as triglycerides in adipose tissue, accompanied by the accumulation of fat and the enlargement of fat cells; some lipid may infiltrate other organs such as the liver and pancreas. Ectopic fat could produce and secrete a variety of metabolic, hormonal, and inflammatory products that produce damage in organs such as the arteries, heart, liver, muscle, and pancreas [3]. Meanwhile, high-fat diet also results to the disorder of gut microbiota and subsequently causes obesity of the host, through changing microbial-derived metabolites, such as reduction in short-chain fatty acids (SCFAs) and bile acids, and production of lipopolysaccharide (LPS) and branched-chain amino acids (BCAAs), which induce glucose and insulin homeostasis imbalance, increase food intake, active proinflammatory responses, and cause an increase of intestinal permeability [4]. Healthy microbiota has great influence on the epithelial barrier functions via the producing short-chain fatty acids (SCFAs) and interactions with innate pattern recognition receptors in the mucosa, driving the steady-state expression of antimicrobial factors [5].

Tea was made from the leaves of *Camellia sinensis*, which is one of the most commonly consumed drinks in the world [6]. Based on the production processing and the variation of polyphenol oxidation, six types of tea with different components can be classified, including green tea, white tea, yellow tea, blue tea (mainly oolong), black tea, and dark tea. Previous studies documented that tea consumption (including tea and its extract) had various positive effects on metabolic disorder [7, 8]. However, different types of tea seemed to have different impacts on lipid metabolism. Reports showed that TPs can affect the central nervous system by through the “microflora–gut–brain axis,” in which the microbiota and its composition determines brain health [9]. A study compared the antiobesity efficiency of different tea types found that white tea, yellow tea, and blue tea increased the carnitine palmitoyltransferase-I (CPT-1) level, while white tea, green tea, and raw Pu-erh tea (a kind of dark tea) decreased the fatty acid synthase (FAS) level [10]. Although efforts had been made, our knowledge of different metabolism regulation effects of tea types and microbiota response to different tea treatments is still limited. Besides, previous studies which using powered tea may influence the proportion of components in tea. To imitate the habit of drinking tea, we neither chose to use purified active ingredients in tea nor did we use powered tea.

Many factors can affect intestinal flora, among which dietary factors have got the most attention due to their effectiveness, simplicity, and low cost [11]. The gastrointestinal tract contains many complex microbes that play significant roles in digestion and metabolism with profound effects on nutrition and health of the host [12]. There are many reports shown that tea polyphenols had the ability to regulate intestinal flora [11]. However, the underlying mechanism is still unknown. In this study, we investigated the effect of six different tea treatments on glucose and lipid metabolism and intestinal flora in mice with high-fat diet and analyzed the potential role of gut microbiota in high-fat diet mice with tea treatments by the way of imitating human-tea-drinking habits.

## 2. Materials and Methods

### 2.1. Animals

Four-week-old C57BL/6J male mice were purchased from the Shanghai SLAC Laboratory Animal Co., Ltd. Four to five mice were kept in one cage. All the mice were maintained under standard laboratory conditions at a temperature of 23°C with 12 h light-dark cycles with free access to food and water. All animal procedures were approved by the Institution Animal Care and Treat Committee at Fudan University. The mice were allowed free access to standard chow diet and water for a week. After a week of adaptation, mice were fed a high-fat diet (HFD) of 60% fat (D12492; Research Diets, USA) for 12 weeks. Control mice still were fed a normal-fat diet (NFD) of 4.5% fat (Purina) for the same period. Mice were randomly and equally divided (7 mice per group) into normal-fat-diet (NFD), high-fat-diet (HFD), yellow tea (HY), dark tea (HB), white tea (HW), green tea (HG), black tea (HR), and blue tea (HT) groups. Mice were divided into 2 groups randomly. One group is treated orally with six types of tea (0.1 ml/10 g/day) and the other group with ddH_2_O (0.1 ml/10 g/day) daily for 6 weeks. Body weight was recorded daily, and blood glucose was measured at 1st and 6th weeks for the 6-week-feeding period. After five weeks of intragastric administration, the mice were scarified. Blood samples were collected at room temperature for three hours and then centrifugation at 3000 rpm for 15 minutes to obtain the serum. The livers and cecum fecal were collected and kept in freezing sterile pipes frozen in liquid nitrogen, then stored at -80°C until used. Our study that was approved by the institutional review board was conducted in accordance with the ethical principles.

### 2.2. Infusion of Tea

Six types of tea were selected in this study listed in Table 1. Mice were treated orally with six types of tea (0.1 ml/10 g/day) or vehicle (autoclaved sterilized water) daily for 6 weeks. Dark tea, white tea, and yellow tea were boiled to make the tea soup (0.1 g/1 ml). Green tea, blue tea, and black tea were brewing with boiled water (0.1 g/ml).

### 2.3. Biochemical Analysis in Serum

The total cholesterol (TC, ab65390, Abcam), triglyceride (TG, ab65336, Abcam), high-density cholesterol (HDL, ab65390, Abcam), and low-density cholesterol (LDL, ab65390, Abcam) levels in serum were measured using the corresponding commercial kits, according to manufacturer's protocol. Insulin in the serum (INS, ab277390, Abcam) was measured using ELISA kits, following the manufacturer's instructions.

### 2.4. Liver Tissue Analysis

The concentrations of malondialdehyde (MDA, ab118970, Abcam), superoxide dismutase (SOD, ab65354, Abcam), IL-6 (ab100713, Abcam), and TNF-alpha (ab100747, Abcam) in the liver were measured using ELISA kits, following the manufacturer's instructions.

### 2.5. Histological Staining

After draining the blood, the liver was soaked in 4% paraformaldehyde solution for more than 24 h. Tissues were then putted it into the hanging basket and dehydrate with gradient ethanol (75%-100%) in order subsequently embedded in paraffin wax. The embedded tissue was sectioned (4 *μ*m), stained with hematoxylin and eosin (H & E), examined by light microscopy (Nikon Eclipse CI, Japan), and photographed.

### 2.6. Real-Time qPCR Analysis

Total RNA from the liver was isolated from liquid nitrogen frozen and ground tissues. The RNA concentration and purity were analysis using the Nanodrop 2000 (Thermo Scientific, MA, USA). The reverse transcription was conducted at 25°C for 5 minutes, 42°C for 30 minutes, and 85°C for 5 seconds. Primers used in this study were designed according to mouse sequence (Table 2). *β*-Actin was chosen as the house-keeping gene to normalize target gene levels. The PCR cycling condition was 40 cycles at 95°C for 15 seconds and 60°C for 60 seconds. The relative expression was expressed as a ratio of the target gene to the control gene using the formula 2^−(∆∆Ct)^.

### 2.7. Microbiota Analysis

The cecal contents were freshly collected and stored at -80°C before extraction. The E.Z.N.A. Stoll DNA Kit (D4015, Omega, Inc., USA) was used for microbial DNA extraction, according to manufacturer's instructions. The V3-V4 region of the 16S ribosomal RNA gene was amplificated using primers 341F (5′-CCTACGGGNGGCWGCAG-3′) and 805R (5′-GACTACHVGGGTATCTAATCC-3′). The amplicon pool was quantified using the Library Quantification Kit for Illumina (Kapa Biosciences, Woburn, MA, USA). High-throughput sequencing was performed using NovaSeq PE250 platform.

Paired-end reads were merged using Fast Length Adjustment of Short reads (FLASH) [13]. Raw data was filtered to generate clean data, using fqtrim (-P 33 -q 20 -w 100 -l 100 -m 5) [14]. Chimeric sequences were removed using VSEARCH [15]. The sequence reads were categorized using the Divisive Amplicon Denoising Algorithm 2 (DADA2) package in R [16]. The SILVA v132 database was used for taxonomically classify features. Alpha and beta diversities were calculated using QIIME2 [17]. Graphs were drawn by R. The LEfSe method was used to obtain significantly differential taxa between groups [18].

### 2.8. Statistical Analysis

All statistical analyses were conducted using the GraphPad Prism 8.0.1 software (GraphPad Software, La Jolla, CA, USA) and RStudio. Multiple groups were compared by analysis of variance (ANOVA). Includes results of weight and blood glucose, ELISA and biochemical analysis. Tukey or Dunn's multiple comparison procedure was used for post hoc comparisons. For nonparametric variables, the Kruskal-Wallis test with Dunn's multiple comparison test was used to assess significance to the differences between groups (R package PMCMR). *p* values < 0.05 were considered statistically significant (∗/#). Data are presented as the mean ± SD.

## 3. Results

### 3.1. Tea Treatments Improve Metabolic Disorder-Related Symptoms in High-Fat Diet Mice

The effects of tea on body weight in mice are shown in Figure 1. Compared with the mice receiving NFD, the final body weight of the HFD group significantly increased (Figure 1(a)). However, tea treatment suppressed the body weight. In addition, different teas revealed varying degrees of effect on inhibiting body weight gain (Figure 1(b)). Notably, the HW, HG, and HT group had a significant decrease on body weight gain.

Lipid profile of mice is also greatly impacted in HFD mice, which is a target to evaluate visceral fat. The value of TC, TG, HDL, and LDL in the HFD group was all higher than that of the control group which indicated successful modeling (Figures 2(a)–2(d)). The content of TC in the liver was significantly decreased by white tea (HW) and black tea (HR) treatments (Figure 2(a)). For TG and HDL levels, the tea groups had no significant difference compared with the HFD group or the NFD group (Figures 2(b) and 2(c)). However, tea did not play a positive role on the concentration of LDL during this experiment (Figure 2(d)).

The liver is one of the tissues that accumulated excessive lipid induced by diet. High-fat diet (the HFD group) significantly increased the liver weight compared with the NFD group (Figure 2(e)). All tea treatments restrained the lipid accumulation in the liver, which reduced the liver weight and liver index compared with the HFD group (Figures 2(e) and 2(f)). Tea treatments of dark tea and white tea even reduced the liver weight of high-fat diet mice to wild-type (Figure 2(e)). The protective effect of tea treatments against liver injury induced by high-fat diet was observed through histopathological analysis. Compared with the NFD group, the HFD group showed visible pathological changes, involving disordered cell arrangement, infiltration of inflammatory cells, and an abundant of lipid droplets (Figure 2(g)). All tea treatments visibly decreased pathological changes in the liver. Taken together, dark tea and white tea had the most powerful function on liver steatosis. However, the liver injury could not be restored by tea, and lipid droplets and disordered cell arrangement still could be observed in tea groups (Figure 2(g)).

Meanwhile, tea supplementation protects against systemic insulin resistance (IR) improving hepatic insulin sensitivity and hyperinsulinemia. Blood glucose after 6 h fasting was significantly reduced in the HY, HB, HW, HG, and HT groups, compared with the HFD group (Figure 2(h)). Along with the decreased blood glucose, the plasma insulin level was also significantly reduced in the HY, HB, HW, and HG groups, with yellow tea (HY) and dark tea (HB) as the most effective treatments (Figure 2(i)). Altogether, these data indicate tea as a good weight-reducing drink for regulations of liver weight and IR.

### 3.2. Tea Treatments Alleviate Major Liver Inflammatory Cytokines and Redox State

As shown in Figures 3(a) and 3(b), the protein expression of IL-6 and TNF-*α* in the liver of the HFD group mice showed a significant increase compared to those of the control group, while the treatment groups had different effect on IL-6 and TNF-*α*'s protein expression. Yellow tea (HY) treatment was most effective in IL-6 protein expression level reduction, which significantly decreased the IL-6 level in high-fat diet mice (Figure 3(a)), while yellow tea, dark tea (HB), and white tea (HW) treatments showed more positive effect in the TNF-*α* regulation, which reduced the level of TNF-*α* in high-fat diet mice to wild-type (Figure 3(b)). Blue tea, green tea, and black tea seemed to have no effect on either in this study.

In order to investigate the ability of various teas to repair oxidative damage in high-fat diet mice, we examined the concentrations of SOD and lipid peroxidation product MDA in the liver. After 18 weeks of high-fat diet, the level of MDA significantly increased in the liver of the HFD group compared with the NFD group (Figure 3(c)). Except green tea treatment (HG), tea treatments significantly reduced the MDA level compared with the HFD group (Figure 3(c)). Yellow tea, dark tea, white tea, and red tea treatments restored the MDA level to wild-type with no significant difference compared with the NFD group (Figure 3(c)). However, the activity of SOD was only significantly increased by yellow tea treatment, which was also observed in the alcoholic fatty liver model mice with black tea, dark tea, and blue tea treatments [19] (Figure 3(d)).

### 3.3. Tea Treatments Affect the Gene Expression Involving Glycometabolism

To understand the metabolic changes that accompanied the phenotype of HFD, we evaluated the expression of key genes involved in the glucose and lipid hepatic metabolism. As Figures 4(a) and 4(b), AMPK*α* was upregulated by green tea on the level of mRNA in the liver (Figure 5(a)). No significant changes were observed among all treated groups of the mRNA level of ACC. Besides, the HB and HW groups had a lower expression of ACC (Figure 5(b)). CPT-1 is the rate-limited enzyme of fatty acid oxidation and had a higher expression in model group (Figure 5(c)). Increased consumption of fatty acids may be due to excessive calorie intake. This phenomenon has been confirmed in population study [1]. The mRNA expression of CPT-1 was upregulated in the HY, HW, HG, HR, and HT groups with statistically significant compared to the NFD group (Figure 5(d)). GAPDH (glyceraldehyde-3-phosphate dehydrogenase) is a key enzyme involved in glycolysis. No obvious regulatory effect on the expression of GADPH was detected among all experiment groups and control groups (Figure 5(e)). For G-6-Pase, there was a significant higher expression in the HY, HB, HW, HG, and HR groups (Figure 5(f)).

### 3.4. Tea Treatments Change Gut Microbial Structure

The structure of gut microbiota was analyzed using 16S rRNA sequencing data. Compared with the NFD group, the HFD group showed significant lower operational taxonomic unit (OTU) number (Figure 4(a)) and alpha-diversity indexes (Figures 4(b) and 4(c)), while tea treatment could not significantly restore diet-induced decreases in OTU number and diversity, with no significant differences between tea treatment groups and the HFD group (Figures 4(a)–4(c)). Compared with other tea, yellow tea (HY) and dark tea (HB) treatments showed better performances in the prevention of obesity-driven dysbiosis (Figures 4(a)–4(c)).

Comparison of microbial structure between groups indicated that diet caused more remarkable changes than tea treatment. However, tea treatment turned the gut microbial structure in HFD mice towards to the structure in NFD mice, as evidenced by species abundance cluster analysis at phylum and genus levels (Figure 4(d) and Figure S1). Results of principal coordinate analysis (PCoA) also showed the same trend. Tea treatment mice clustered partially apart of HFD mice, suggesting important changes in gut microbiota induced by tea treatment (Figure 4(e)). According to PCoA, yellow tea (HY) treatment showed the most positive effect on HFD mice, with values clustered between HFD and NFD groups (Figure 4(e)).

To investigate composition changes of gut microbiota among groups, we compared relative abundances of taxa at phylum and genus levels. At the phylum level, the relative abundance of Firmicutes was only significantly changed between HG and NFD (Figure 6(a)), while the decrease in Bacteroidetes and the increase in Proteobacteria and Deferribacteres were common in the HFD and tea treatment groups (Figure 6(a)). Part of the decrease in Bacteroidetes could be explained by the significant reduction in unclassified Muribaculaceae. Tea supplement did not change the decrease trend of Bacteroidetes in obesity mice. Green tea (HG) and black tea (HR) did not reduce the abundance of Bacteroidetes significantly as compared with NFD (Figure 6(a)), which showed a better performance than other tea. Firmicutes did not significantly changed in HFD and tea treatment groups as compared with NFD, except in the HG group.  Figure 6(b) shows that in the HFD group, the reduction of Spirulina species led to the reduction of most Firmicutes. Caused by the reductions in both Firmicutes and Bacteroidetes, the Firmicutes/Bacteroidetes ratio had no significant change between HFD and NFD (Figure S2A), while the Firmicutes/Bacteroidetes ratio significantly increased in HY compared with NFD, which was caused by the significantly decrease in Bacteroidetes in the HY group. The most of increment in Proteobacteria could be explained by the significant increment in *Bilophila* at the genus level (Figure 6(b)). Tea supplement slightly prevented the increase trend of *Bilophila* in obesity mice, with yellow tea (HY) as the best treatment (Figure 6(b)). At the genus level, tea treatment significantly changed the relative abundance of *Lachnospiraceae_unclassified* (increased in HY, HB, and HG) and *Alistipes* (reduced in HG) as compared with HFD. The relative abundance of *Bifidobacterium* was extremely low in all groups (Figure S2B), which also appeared in previous study [20]. Red tea treatment significantly restores the decrement of *Bifidobacterium* in obesity mice, and white tea treatment induced a slightly but not significant increase in *Bifidobacterium* (Figure S2B).

The linear discriminant analysis (LDA) effect size (LEfSe) approach revealed specific taxa in different groups. Compared with HFD mice, yellow tea (HY) treatment induced the most similar discriminative taxa pattern to the pattern of NFD (Figures 6(c) and 6(d)). The LEfSe distinguished HY from HFD by the higher abundance of Clostridiales order, *Lachnospiraceae_unclassified* spp., Lachnospiraceae family, and *Helicobacter_unclassified* spp. and the lower abundance of Bacteroidales order, *Bilophila* genus, Desulfovibrionales family, Rikenellaceae family, and *Alistipes* genus (Figure 6(d) and Figure S3). The higher abundance of Lachnospiraceae and Clostridiales also appeared in NFD as compared with HFD, and the lower abundance taxa in HY showed a same trend in NFD (Figure 6(c)). Bacteroidetes was identified as a lower tax on in HY, which was caused by a lower abundance of *Alistipes* compared with HFD (Figures 6(b)–6(d)), while the higher abundance of Alistipes in HFD not only appeared in the comparison with HY but also in the comparison with NFD (Figure 6(d)). So, the decrease in Bacteroidetes in the LEfSe result of the HY group did not mean that yellow tea aggravated the HFD-driven dysbiosis.

Compared with the HFD group, the higher abundance of *Lachnospiraceae_unclassified* spp. commonly appeared in tea treatment groups except the HT group (Figure S3). Besides, tea supplement also induced the lower abundance of Bacteroidales order (HY, HB, and HW), Rikenellaceae family (HY, HB, HW, HR, and HG), and *Alistipes* genus (HY, HB, HW, and HG). White tea (HW) supplement reduced the abundance of *Ruminiclostridium_unclassified* spp. (Figure 6(b) and Figure S3). Although Helicobacter was identified by LEfSe as the higher discriminative taxon in tea treatment groups, the relative abundance of it had no significant difference between all groups (Figure 6(b)). So we considered that tea treatment regulated the abundance of *Lachnospiraceae_unclassified* spp., Clostridiales order, Bacteroidales order, Rikenellaceae family, *Alistipes* genus, and *Ruminiclostridium_unclassified* spp. According to LEfSe, yellow tea, dark tea, white tea, and green tea supplements could regulate the gut microbiota structure in HFD mice, while blue tea supplement had no significant improvement.

## 4. Discussion

For overweight or obese patients, losing weight may bring unexpected benefits [21]. Tea has been proved to be a good fat-reduction drink, which was widely confirmed in both mice and human subjects [7, 22, 23], and was also found in the present study. According to the literature, we summarized three major mechanisms of suppressing fat accumulation involving tea: (1) inhibiting adipogenesis; (2) decreasing absorption of lipids and proteins by tea constituents in the intestine, thus reducing calorie intake or increasing the fecal energy excretion; and (3) downregulating the gene expression of lipogenic enzymes and related transcription factors and upregulating the mRNA level of fat *β*-oxidation genes in the liver, skeletal muscle, and adipose tissues [24, 25]. AMP-activated protein kinase- (AMPK-) related signal pathway plays a major role in regulating cellular energy metabolism balance. Activated AMPK has been shown to decrease the expressions or activities of acetyl-CoA carboxylase (ACC) (for fatty acid synthesis) and carnitine palmitoyltransferase-1 (CPT-1) (for fatty acid *β*-oxidation). Studies have found that green tea can increase the expression of genes related to lipid oxidation, preventing the accumulation of liver fat through the activation of AMPK [26], which was confirmed in our subject. Also, the mRNA expression of AMPK*α* was increased of HFD mice via 6-week treatment of green tea. It seems that the function of inhibiting obesity of green tea is by regulating the AMPK/CTP-1 signal pathway. Although the same conclusion also documented with blue tea [8], the expression of AMPK*α*, ACC, and CTP-1 determined by RT-qPCR had on significant change compared to HFD group which may due to the different tea selection. However, a comparative study of black, green, blue, and white teas shows that blue tea most effectively blocked weight gain [23], which is consistent with our results. Rather than directly regulating AMPK gene expression, white tea intervention restored the suppressed expression of p-AMPK protein in type 2 diabetes C57BL/6 mice [27]. However, the content of p-AMPK protein did not increase in ICR mice fed with high-fat diet [10]. The mechanism of suppress weight of white tea and blue tea should continue to be explored. Dark tea and white tea exhibited the best effect on liver weight and liver index, and the pathological sections further verify this conclusion, which may result of the lowest mRNA expression of ACC.

Fasting blood glucose comes from endogenous glucose, and the liver is the source of endogenous glucose [28]. Elevated fasting blood sugar is the result of liver insulin resistance. Our results suggested that tea can alleviate hyperglycemia and hyperinsulinemia and improve the sensitivity of insulin in liver. However, the results of RT-qPCR showed that tea upregulates the mRNA expression of G-6-Pase, a gluconeogenesis-related enzymes in the liver. The rise of Lachnospiraceae was consistent with the G-6-Pase expression (Figure S1 and Figure 1(h)). Since propionate is a secretion of Lachnospiraceae, it is a prerequisite for hepatic gluconeogenesis and improves the balance of glucose and insulin [4]. The upward movement of G-6-Pase may because of a dramatic drop in blood sugar.

Tea polyphenols are generally recognized as strong antioxidants because of its special molecular structure, and their antioxidant action has been suggested to contribute to the alleviation of metabolic syndrome. Tea flavanols (such as catechin and epicatechin) inhibited the growth of several pathogens and have an inhibitory effect on the growth of symbiotic anaerobes [9]. EGCG, an active polyphenolic catechin of tea, which is the most abundance of green tea, plays a major role in the role of antioxidant. Nevertheless, studies from in vitro have increasingly mentioned that green tea extract and EGCG seem to have a dose effect and are cytotoxic at high concentration [29]. The amount of tea patients takes every day might be different dose. The highest content of MDA in the green tea groups is possibly due to the toxicity of polyphenols caused by high concentrations. Compared with the other five types of tea, yellow tea can simultaneously restrain the peroxidation of fatty acids and stimulate the activity of SOD to resist the oxidative stress caused by a high-fat diet.

Tea treatment had positive effects on dysbiosis drove by the high-fat diet. Based on the result of PCoA and LEfSe, yellow tea treatment showed the best performance, which partly recovered the disorder of model mouse microbiota. As for the Firmicutes/Bacteroidetes ratio, yellow tea treatment was the only significantly increased treatment compared with wild type. In the HY group, the increment of Firmicutes/Bacteroidetes ratio is relatedto the significant decrease of Bacteroidetes, and the decrease of Bacteroidetes is related to the decrease in *Alistipes*, according to LEfSe. Although the Firmicutes/Bacteroidetes ratio is a biomarker of obesity-driven dysbiosis [30], the increase of this ration in HY may not mean that yellow tea increased the microbiota disorder, as *Alistipes* also decreased in wild-type. The human gut microbiota study also showed no significant correlation between the abundance of Firmicutes and obesity or between the abundance of Bacteroidetes and obesity [31].

The decrement of unclassified Lachnospiraceae in HFD mice was significantly restored by yellow tea, white tea, and green tea treatments. Lachnospiraceae members are short-chain fatty acid propionate producers and microbiota composition modulator in gut [32]. Unclassified Lachnospiraceae members enrich in the gut microbiota of centenarians in China and Italy [33, 34]. Therefore, the increase in unclassified Lachnospiraceae could be a signature of positive effects tea treatment provided, which turned the high-fat diet microbiome towards a healthy and longevity microbiome [35]. Along with the increase in unclassified Lachnospiraceae, inflammatory cytokines (involving IL-6 and TNF-alpha) also significantly reduced by yellow tea and white tea treatments, while the content of inflammatory cytokines had no decrease in the blue tea group compared with obesity mice. This result suggests the negative relationship between Lachnospiraceae and inflammation, which is in line with previous study in mice [32]. Previous studies have shown that HFD can significantly alter the composition of gut microbes [36]. HFD might lead to increased hepatic retention of hydrophobic bile acids, which are significantly associated with changes in intestinal microorganisms [37].

The increment of *Alistipes* in HFD mice was regulated by yellow tea, dark tea, white tea, and green tea treatments, and green tea treatment significantly prevented the *Alistipes* increment. *Alistipes* members are putrefactive microbes in gut, which relate to the fermentation of amino acid and production of short-chain fatty acids [38]. The increase of *Alistipes* in gut relates to the obesity or high-sugar food supplement [20, 39]. Yellow tea and white tea supplements not only reduced the *Alistipes* but also significantly reduced the level of TC and HDL in HFD mice. This positive correlation between *Alistipes* and disorders of glucose and lipid metabolism is also consistent with the results reported by Song et al. [20].

However, the effects of tea treatment were limited, compared with the strong alters caused by diet. The animal-based diet (high-fat and high-protein) can rapidly increase the abundance of bile-tolerant bacteria (*Bilophila*, *Alistipes*, and *Bacteroides*) and decrease the abundance of polysaccharide-metabolic Firmicutes in human gut microbiota [38]. The same trend also appeared in the gut microbiota of HFD mice with 60 kcal% fat diet (lard/soybean oil = 9.8). Yellow tea treatment reduced the abundance of *Alistipes* and *Bacteroides* in model mice to the level of them in wild-type (the relative abundance of *Alistipes* was 2.47% in NFD and 2.17% in HY; the relative abundance of *Bacteroides* was 0.55% in NFD and 0.55% in HY), along with the increase in Firmicutes. However, the abundance of *Bilophila* increased in all tea treatment groups, which shows the limitation of tea treatment in microbial regulation. Yellow tea treatment also showed the best performance in the reduction in *Bilophila*.

Green tea, especially when consumed in large amounts on an empty stomach, is known to cause irritation in the gastrointestinal system. Black tea is considered to be milder (less irritating), but the beneficial health effects are weaker [25]. Pu-erh tea and blue tea are considered effective in many studies, though there are also inconsistent conclusions. The health effects of white tea and yellow tea lack more experimental evidence. Although the beneficial effects of tea on glucometabolic and intestinal flora have been found in human and animal experiments, and our experiments have also found some positive functions, it is obviously undesirable to try to rely solely on daily supplements of tea to treat diseases. Perhaps, long-term treatment will achieve the effect of “one plus one greater than two,” which will require more experiments to prove it.

## 5. Conclusion

Taken together, these results revealed that tea can inhibit the weight gain and attenuate hepatic steatosis and insulin resistance. The anti-inflammatory and antioxidant effects of yellow tea, white tea, and dark tea are salient. The underlying mechanism seems different among six types of tea. Green tea significantly upregulated p-AMPK and CPT-1, probably because that green tea inhibits obesity by increasing energy expenditure and fatty acid oxidation. Dark tea and white tea exhibited the best effects on liver weight and liver index which may result from the lowest mRNA expression of ACC. Yellow tea treatment was the best on the disorder of intestinal flora. The unclassified Lachnospiraceae and *Alistipes* in HFD mice were regulated by yellow tea, white tea, and green tea treatments. We did not find significant results about black tea and blue tea in the RT-q PCR experiment in the present study. This study demonstrated that various tea drinking has beneficial effects for HFD-related metabolic disorders.

## Figures and Tables

**Figure 1:** Tea treatments inhibited the body weight in high-fat diet mice: (a) body weight; (b) body weight gain. Data were expressed as mean ± SD and assessed Kruskal-Wallis test with Dunn's multiple comparison test (*n* = 7), ^∗∗^*p* < 0.01 compared with the HFD group.

**Figure 2:** Tea treatments improve metabolic disorder-related symptoms in high-fat diet mice: (a) serum TC concentration; (b) serum TG concentration; (c) serum HDL concentration; (d) serum LDL concentration; (e) liver index; (f) liver weight; (g) HE staining of liver; (h) blood glucose; (i) serum insulin content. Data were expressed as mean ± SD. (a–f, i) Kruskal-Wallis test with Dunn's multiple comparison test, (h) analysis of variance (ANOVA), and Tukey multiple comparison (*n* = 7), ^∗^*p* < 0.05, ^∗∗^*p* < 0.01 compared with the HFD group. ##*p* < 0.01 compared with the NFD group.

**Figure 3:** Tea treatments alleviate major liver inflammatory cytokines and redox state in liver: (a) liver IL-6; (b) liver TNF-alpha content; (c) liver MDA content; (d) liver SOD activity. Data were expressed as mean ± SEM. (a–c) Analysis of variance (ANOVA) and Tukey multiple comparison (*n* = 7). Differences of data (d) were assessed by Kruskal-Wallis test with Dunn's multiple comparison test, respectively (*n* = 7). ^∗^*p* < 0.05, ^∗∗^*p* < 0.01 compared with the HFD group. #*p* < 0.05, ##*p* < 0.01 compared with the NFD group.

**Figure 4:** Tea treatments modify the structure of the cecal microbiota in high-fat diet mice: (a) OTU number; (b) Shannon index (at OTU level); (c) Simpson index (at OTU level); (d) taxa abundance cluster analysis at the phylum level. (e) Principal coordinate analysis (PCoA) on Bray-Curtis distance matrix. (a–c) Kruskal-Wallis test with Dunn's multiple comparison test. *N* = 7 per group. #*p* < 0.05, ##*p* < 0.01, compared with the NFD group; ^∗^*p* < 0.05, ^∗∗^*p* < 0.01, compared with the HFD group.

**Figure 5:** Tea treatments affect the gene expression involving glycometabolism of the liver measured by RT-qRCR: (a) AMPK*α*; (b) ACC; (c) CPT-1; (d) GADPH; (e) G-6Pase. Differences of data were assessed by Kruskal-Wallis test with Dunn's multiple comparison test (*n* = 7). Data were expressed as mean ± SD. ^∗∗^*p* < 0.01 compared with the HFD group.

**Figure 6:** Tea treatments modify the composition of the cecal microbiota in high-fat diet mice. Relative abundance of taxa at (a) phylum and (b) genus level. (c) Linear discriminant analysis (LDA) of differentially abundant taxa between the model group and the control group. (d) LDA of differentially abundant taxa between the model group and the yellow tea treatment group. (a, b) Kruskal-Wallis test with Dunn's multiple comparison test. #*p* < 0.05, ##*p* < 0.01, compared with the NFD group; ^∗^*p* < 0.05, ^∗∗^*p* < 0.01, compared with the HFD group.

**Table 1:** Characteristics of included studies.

Type	Name	Manufacture origin	Way of make soup	Group
Dark tea	Golden fungi	Qiyan, Hunan province	Boiled	HB
White tea	Old eyebrow	Fuding, Fujian province	Boiled	HW
Yellow tea	Golden buns	Jiangkou, Guizhou province	Boiled	HY
Green tea	Green pearls	Meitan, Guizhou province	Brewed	HG
Blue tea	Titkuanyim	Anxi, Fujian province	Brewed	HT
Black tea	Yunnan red	Yongping, Yunnan province	Brewed	HR

**Table 2:** Nucleotide sequences of primers.

Gene	Forward sequence (5′-3′)	Reverse sequence (5′-3′)
AMPK*α*	CTCAGGAAGGCTGTATGCGG	ACG GTTGAGATACTCCGGGAT
ACC	ATGCTATTTCTTTGTTTGGTCGT	CCCAGCACTCACATAACCAAC
CPT-1	CTTCAATACTTCCCGCATCCCT	AGCAGCCTCCCGTCATGGTA
GAPDH	TCATCTCTGCCCCCTCTGCT	CGACGCCTGCTTCACCACCT
G-6-Pase	GTAGAATCCAAGCGCGAAAC	TCTGTCCCGGATCTACCTTG

## Data Availability

All raw sequences from 16S rRNA gene-based analysis have been deposited in the public European Nucleotide Archive server under accession number PRJNA742157.

## Supplementary Materials

Supplementary Materials Figure S1: taxa abundance cluster analysis at the genus level. Figure S2: (A) Firmicutes to Bacteroidetes (F/B) ratio (relative abundance of Firmicutes/relative abundance of Bacteroidetes). (B) The relative abundance of Bifidobacterium. Kruskal-Wallis test with Dunn's multiple comparison test. #*p* < 0.05, ##*p* < 0.01, compared with the NFD group. Figure S3: LDA scores of differentially abundant taxa between the HFD group and other groups using the LEfSe method.
